The article "Monitoring System-Based Flying IoT in Public Health and Sports Using Ant-Enabled Energy-Aware Routing" was retracted in 2023. Reasons: unreliable results or conclusions; concerns about the data; concerns about the peer review; concerns about the citations.

# Monitoring System-Based Flying IoT in Public Health and Sports Using Ant-Enabled Energy-Aware Routing

**DOI:** 10.1155/2021/1686946

**Published:** 2021-07-01

**Authors:** Inam Ullah Khan, Muhammad Abul Hassan, Mohammad Dahman Alshehri, Mohammed Abdulaziz Ikram, Hasan J. Alyamani, Ryan Alturki, Vinh Truong Hoang

**Affiliations:** ^1^Department of Electronic Engineering, School of Engineering and Applied Sciences, Isra University, Islamabad, Pakistan; ^2^Department of Computing and Technology, Abasyn University, Peshawar 25000, Pakistan; ^3^Department of Computer Science, College of Computers and Information Technology, Taif University, Taif 21944, Saudi Arabia; ^4^Computer Science Department, University College in Al-Jamoum, Umm Al-Qura University, Makkah, Saudi Arabia; ^5^Department of Information Systems, Faculty of Computing and Information Technology in Rabigh, King Abdulaziz University, Jeddah, Saudi Arabia; ^6^Department of Information Science, College of Computer and Information Systems, Umm Al-Qura University, Makkah, Saudi Arabia; ^7^Department of Information Technology Specialization, FPT University, Hoa Lac High Tech Park, Hanoi, Vietnam

## Abstract

In recent decades, the Internet of flying networks has made significant progress. Several aerial vehicles communicate with one another to form flying ad hoc networks. Unmanned aerial vehicles perform a wide range of tasks that make life easier for humans. However, due to the high frequency of mobile flying vehicles, network problems such as packet loss, latency, and perhaps disrupted channel links arise, affecting data delivery. The use of UAV-enabled IoT in sports has changed the dynamics of tracking and working on player safety. WBAN can be merged with aerial vehicles to collect data regarding health and transfer it to a base station. Furthermore, the unbalanced energy usage of flying things will result in earlier mission failure and a rapid decline in network lifespan. This study describes the use of each UAV's residual energy level to ensure a high level of safety using an ant-based routing technique called AntHocNet. In health care, the use of IoT-assisted aerial vehicles would increase operational performance, surveillance, and automation optimization to provide a smart application of flying IoT. Apart from that, aerial vehicles can be used in remote communication for treatment, medical equipment distribution, and telementoring. While comparing routing algorithms, simulation findings indicate that the proposed ant-based routing protocol is optimal.

## 1. Introduction

According to the reports, the Flying Ad-Hoc Network (FANET) is a recently emerged area in sensor networks with a decentralized communication mechanism. However, because of ad-hoc dynamics, each node collects data and sends it to the base station via a backbone aerial vehicle. In the last couple of years, flying vehicles have evolved and operated in every aspect of life, such as traffic monitoring, agricultural monitoring, border surveillance, smart cities, and, more importantly, limited-time rescue operations. Drones are deployed in operation areas to collect data. However, aerial vehicles are categorized into small and large sizes. In contrast, small-size UAVs have an extra edge over large-size UAVs because of their versatile light-weight behavior, flexibility, low altitude flying, easy installation, and low hardware cost. Multiple UAV networks have been preferred over single ones because of (i) efficiency, (ii) scalability, and (iii) survivability and accuracy. In comparison with single UAV's, a multibackbone aerial network has encountered long-range surveillance.

The article "Monitoring System-Based Flying IoT in Public Health and Sports Using Ant-Enabled Energy-Aware Routing" was retracted in 2023. Reasons: unreliable results or conclusions; concerns about the data; concerns about the peer review; concerns about the citations.

The flying ad hoc network has an extra edge over its predecessors because of its low hardware cost, ease of deployment, autonomy, and availability in every situation. Aerial vehicles are tolerable enough to adopt any direction in three-directional space, making it more feasible for time-limited rescue missions [1]. Three-dimensional mobility of flying things made topological permutations very high, limiting limitations in terms of energy, insufficient bandwidth, and robust computations in communication links. The bandwidth of aerial vehicles is about 30–460 km/h [2], which in return causes routing and disconnection problems in flying networks. Different routing protocols are applied to encounter the routing problem in FANETs. However, high mobility patterns in aerial networks need novel energy-efficient routing techniques. In addition, aerial vehicles are interconnected with wireless technology, e.g., IEEE 802.15.4, as shown in Figure 1. In this figure, each flying vehicle monitors an assigned geographical area which establishes a personalized UAV network.  Table 1 discusses the advantage of the multi-UAV network over a single aerial vehicular network. Furthermore, Figure 2 explains the applications based on single UAV to monitor and send data to a base station, while Figure 3 depicts a proposal for connecting two cities using a multi-UAV framework. Mobility models also enhance the utilization of network resources with accurate implementation of routing protocols in a network.

Flying IoT will be designed to monitor athletes in motion during international games. Drones connected to the Internet of things are referred to as Flying IoT, which will reshape player tracking and reduce the risk of injury. This transformation will produce optimum results by incorporating data collection through aerial vehicles. They will improve efficiency, real-time player experience, and new revenue-generating opportunities in sports. Flying IoT has many benefits, including the ability to reach heights, produce high-quality images at a low cost, and respond quickly in any scenario [3].

The article "Monitoring System-Based Flying IoT in Public Health and Sports Using Ant-Enabled Energy-Aware Routing" was retracted in 2023. Reasons: unreliable results or conclusions; concerns about the data; concerns about the peer review; concerns about the citations.

The major contribution in this research article is as follows.

- IoT-based UAVs are used to maximize the quality of service/experience
- The ant-inspired routing protocol is deployed in the area of flying ad hoc networks
- The boundless area mobility model is introduced in the study of the Internet of flying vehicles
- Flying network is analyzed using parameters that include throughput, network utilization, packet delivery ratio, packet drop count, packet loss, and end-to-end delay
- Flying IoT is utilized in the field of sports and health care for monitoring

The rest of the article is structured with Section 1, which consists of the paper Introduction.  Section 2 is composed of brief literature with past data about the problem. Similarly, routing in flying IoT is incorporated in Section 3 also.  Section 4 represents the proposed model.  Section 5 demonstrates the simulation environment. The performance graphs and results are discussed in Section 6. Results and discussion are explained in Section 7. The overall analysis and future direction are discussed in Section 8.

## 2. Literature Survey

The flying ad-hoc network is a subset of the mobile ad-hoc network with some special features as discussed in Section 1; with all these benefits, it also inherits the routing problem due to its rapid changing topology [3]. 3D mobility of flying things enabled expanding of the geographical area which helps in surveillance of the large area by a single UAV. Among other limitations, one of the key problems which must be addressed is lack of specialized routing protocols on the industrial level in the field of flying ad hoc networks [4]. Therefore, classification of aerial networks routing protocols is in the development phase; due to that, FANETs relay on traditional MANET routing protocols [5, 6]. The OPEN routing protocol is a designed novel strategy which is based on (i) residual energy, (ii) node density, and (iii) distance from its neighbors; these metrics are used for electing cluster head (CH) [7]. In [8], authors tested the optimal ant-based distance protocol. Primary metrics are used for the analysis of other routing protocols in the simulation-based environment. The ant-based routing protocol faces flat and hierarchical network topology problems. Due to fast-changing nature, the UAV network is having issues related to routing links failures, disruptions, and signal jamming [9]. Flying ad hoc networks are having different mobility models, nodes' position, and radio frequency in comparison with other areas which include MANETS and VANETS. Wireless communication technologies are utilized to connect nodes with base stations in different fields [10].  Figure 4 describes the brief study of different routing protocols in the newly emerged field known as Internet of flying networks.

The article "Monitoring System-Based Flying IoT in Public Health and Sports Using Ant-Enabled Energy-Aware Routing" was retracted in 2023. Reasons: unreliable results or conclusions; concerns about the data; concerns about the peer review; concerns about the citations.

COVID-19 has increased the use of flying IoT in general. China has deployed drones for crowd monitoring in order to maintain social distance. In addition, several European countries are using unmanned aerial vehicles (UAVs) for announcements or broadcasting in order to take appropriate actions [11]. Agricultural drones may be used to spray disinfectants in order to stop the transmission of a deadly virus. Drones, on the contrary, can be used to deliver medicine quickly and reduce the burden on hospitals [12].

When using IoT-based drones, live sport video streaming is a great challenge. End users need high-quality video experience to capture entertaining scenes, which can be easily achieved using fog networking and UAVs [13]. Aerial IoT is used in a cycling race to propose a novel approach for accuracy optimization using machine learning to train the model [14].

The use of flying IoT in healthcare would revolutionise the world. Aerial IoT can be used to keep track of athletes' fitness when they are competing. However, using routing protocols in the field of healthcare will transform the dynamics of communication. For this purpose, ant-inspired routing, AOMDV, DSDV, DSR, M-DART, and ZRP are implemented to improve channels/links. Therefore, Table 2 discusses latest data survey about routing protocols in UAV-assisted networks.

## 3. Routing in Flying IoT

Flying ad hoc networks are referred to Internet of drones where flying things are connected with land station. Among the aerial nodes, routing plays an important role to find the optimal path from the source to the destination. Demand of unmanned aerial vehicles, while integrating with smart cities needs some basic requirements in routing; for instance, adaptability, scalability, residual energy, delay, and bandwidth complete the network study of aerial vehicles. Routing in flying things depends upon distance, angle of arrival, path lifetime, and node localization to make decisions on right time. Mobile movements of nodes in flying ad hoc networks consist of key steps which include route discovery, broadcasting, selecting path, and link maintenance. Apart from routing in IoT-based networks, security must be ensured [25].

The article "Monitoring System-Based Flying IoT in Public Health and Sports Using Ant-Enabled Energy-Aware Routing" was retracted in 2023. Reasons: unreliable results or conclusions; concerns about the data; concerns about the peer review; concerns about the citations.

Classifications of routing protocols in flying IoT are mentioned below.

### 3.1. Proactive

The word proactive is made of two words pro and active which means storing and maintaining data packets in routing tables to facilitate aerial networks.

### 3.2. Reactive

The reactiveness can be only achieved in multiple flying vehicles in order to transmit data packets when needed. While using reactive strategies, the overhead problem can be easily reduced.

### 3.3. Hybrid

Hybridization is the process of combining two or more features to formulate optimal technique. In addition, both proactive and reactive natures of routing construct the hybrid algorithm.

### 3.4. Bio-Inspired

The techniques which can be simulated by the behaviour of animals, ants, fish, or birds to find the optimal solution in routing are known as bio-inspired.

## 4. Proposed Approach (AntHocNet for Flying Ad Hoc Networks)

Quality of experience-based AntHocNet routing for flying networks is proposed. QoE-based AntHocNet is working on the basic concept of ant colony optimization. Quality of experience is evaluated using different metrics which include throughput, network utilization, packet delivery ratio, packet drop count, packet loss, and end-to-end delay.  Figure 5 represents ant behavior to find the optimal path from the source to the destination. Ant-based reinforcement works on pheromone modeling to choose the route for flying vehicles.

The approach “AntHocNet” [26] is a hybrid algorithm having both reactive and proactive components. Communication process is very important during the whole method for searching food by ants where on-demand events are used. However, maintaining the path and updating pheromone table are performed to control data packets in flying networks. The iterative random sampling mechanism is used to collect routing data packets to enhance adaptability in dynamic flying networks. By deploying ant-inspired technique in flying ad hoc networks, it can help to boost up overall life time and decision-making.

This novel algorithm consists of five main steps which are as follows:

- Initial solution
- Making decision in a centralized way
- Pheromone concentration
- Reinforcement learning or pheromone update
- Pheromone evaporation

The proposed hybrid scheme AntHocNet initializes data session to launch reactive forward ants for searching multiple routes. Also, backward ants are used to maintain the path. Link failure data packets are broadcast, which helps in removal of transmission errors. Pheromone is a watery liquid that will have a high concentration if the number of ants on that trail increases. Also, the process of reinforcement is incorporated that it allows ants to learn from the surrounding environment. Else, if the ants' moment will be very low on the specific path, then pheromone evaporation occurs.

The article "Monitoring System-Based Flying IoT in Public Health and Sports Using Ant-Enabled Energy-Aware Routing" was retracted in 2023. Reasons: unreliable results or conclusions; concerns about the data; concerns about the peer review; concerns about the citations.

In addition, the working flowchart of AntHocNet is mentioned in Figure 6.

## 5. Simulation Environment

Simulation setup consists of thirty flying vehicles and one ground station. The whole study is performed by using network simulator-2. The boundless area mobility model is deployed on three-dimensional topology having 1000 m area for *x*, *y*, and *z* axes. The time exercised for the experimentation was around 180 seconds where constant bit rate data packets are employed as traffic type. The UAV network topology is presented in Figure 7.

## 6. Performance Graphs

In this section, we discuss the results' performance using graphs as shown in the following.

Evaluating routing techniques by using the throughput study is described in Figure 8. The learning of throughput analysis is estimated by levels which include minimum, maximum, average, and standard deviation. The ant-simulated routing algorithm illustrates optimal received data packets per unit time in comparison with other routing schemes.

The packet delivery ratio is to investigate data packets on two metrics which will be either packet sent or packet received.  Figure 9 describes routing schemes such as dynamic source routing, where thirty thousand plus data packets are sent by utilizing the method of broadcasting but very less web of information are received. However, ant-based routing manifests balanced results in contrast with DSDV, M-DART, AOMDV, and zone routing protocol.

As the number of data packets is dropped, it causes huge impact on network lifetime. In addition, the zone routing scheme is a hybrid learning mechanism having both proactive and reactive approaches. Dividing the topological structure in different zones or clusters easily reduces overhead issues inside the flying networks. Therefore, AntHocNet is based on the fundamental concept of ants locating the shortest path by using the pheromone update method which improves the energy level in unmanned aerial vehicles. In Figure 10, routing algorithms such as AntHocNet and ZRP represent better simulation results by estimating the number of packet drop.

During data transmission in flying networks, packet loss occurs due to having bugs.  Figure 11 shows routing protocols and number of packets where AntHocNet is having desired results in terms of packet loss in comparison with other contemporary algorithms.

In IoT-based aerial vehicles, delay can be caused, while retransmitting data packets across the multi-UAV networks. Calculating average end-to-end delay requires data packet length to reach the destination in the defined time frame.  Figure 12 describes the ant routing (AntHocNet) is having very less end-to-end delay from the source to the target.

The article "Monitoring System-Based Flying IoT in Public Health and Sports Using Ant-Enabled Energy-Aware Routing" was retracted in 2023. Reasons: unreliable results or conclusions; concerns about the data; concerns about the peer review; concerns about the citations.

Network utilization is the maximum capacity of data transfer across the network.  Table 3 shows the network utilization study to perform experimentation by using different routing protocols. A novel technique called standard deviation is used to offer greater depth of study by calculating the average or mean.

## 7. Results and Discussion

AntHocNet finalizes to generate both proactive and reactive strategies which learn from the system. Ant routing has been shown to be a suitable solution for flying ad hoc networks due to AntHocNet's self-organizing nature, which demonstrates less tendencies toward packet loss, whereas the packet drop ratio improves quality of service in flying networks. Similar effects are claimed in simulation having less packet drop count. Network scalability can be achieved in aerial vehicles by boosting network throughput. On the contrary, ant-based routing simulates throughput and average end-to-end delay, while simulating with other conventional algorithms. As the paper discusses, the implementation of routing-related monitoring in health care and sports will improve the quality of service in flying networks.

## 8. Conclusions

IoT-based routing plays an important role in the field of flying ad hoc networks. Due to mobile pattern wireless communication technologies [27], deployment allows easy access to aerial vehicles with the base station. The best practice is to use flying IoT in health care and sports. For optimal communication, routing protocols can be used in IoT-based drone networks. Aerial networks require secure channels for transmitting data packets using the routing protocol from one location to another. A novel evolutionary computational algorithm, “AntHocNet,” is introduced in the field of the Internet of flying networks. The ant-inspired technique is evaluated by comparing it with traditional routing protocols, including DSR, ZRP, M-DART, DSDV, and AOMDV. The suggested solution differs from baseline protocols due to certain key features such as learning from the environment, convergence, loop-free, localization, and quality of service. The boundless area mobility model is used in the simulation, which helps to improve reinforcement learning in flying networks. Other mobility model deployment in the field of UAVs would be a valuable addition in the future.

## Figures and Tables

**Figure 1:** Personalized UAV network applications in health care.

**Figure 2:** Single UAV monitoring-based applications.

**Figure 3:** Multi-UAV's connectivity in two different cities.

The article "Monitoring System-Based Flying IoT in Public Health and Sports Using Ant-Enabled Energy-Aware Routing" was retracted in 2023. Reasons: unreliable results or conclusions; concerns about the data; concerns about the peer review; concerns about the citations.

**Figure 4:** Routing protocols for Internet of flying networks.

**Figure 5:** Working of ant colony optimization.

**Figure 6:** Flowchart of AntHocNet.

**Figure 7:** Aerial network topology for UAVs.

**Figure 8:** Throughput analysis.

**Figure 9:** Packet delivery ratio.

**Figure 10:** Packet drop count.

**Figure 11:** Packet loss.

**Figure 12:** Average end-to-end delay.

**Table 1:** Multiple and single aerial vehicles.

Feature	Single FANET-UAV network	Multiple FANET-UAV networks
Failure impact of network	Very high	Very low; other nodes replace the failed ones
Scalability	Limited	High
Survivability	Low	High
Speed of mission	Slow	Very fast
Cost	Medium	Low
Bandwidth	Needed	High
Communication medium	Antenna	Omni-directional
Control complexity	Low	High
Coordination on failure	Low	High

**Table 2:** Latest literature about routing protocols.

Ref.	Routing protocol	Prediction	Connectivity	Exploration	Efficient use of energy	Rapid action against abrupt changes	Network application
[15]	Energy-efficient Connectivity-aware Data Delivery (ECaD) routing algorithm	Available	Available	Available	Available	Not available	Flying ad hoc networks
[16]	Parrot: predictive ad-hoc routing	Available	Not available	Available	Not available	Not available	UAV-aided networks
[17]	ARdeep: adaptive and reliable routing protocol with deep learning	Available	Available	Available	Available	Not available	Mobile robot networks
[18]	QMR	Available	Not available	Available	Available	Available	FANETs
[19]	FLRLBR	Available	Available	Available	Available	Not available	FANETS
[20]	QAGR	Available	Not available	Available	Not available	Not available	FANETs
[21]	Adaptive Q-routing with Random Echo and Route Memory (AQRERM)	Available	Not available	Available	Not available	Not available	FANETs
[22]	Delayed Q-routing (DQ-routing)	Available	Not available	Not available	Available	Not available	FANETs
[23]	Poisson's probability-based Q-routing (PBQ-routing)	Available	Available	Available	Not available	Not available	FANETs
[24]	Traffic-aware Q-network enhanced routing protocol based on GPSR (TQNGPSR)	Available	Available	Available	Not available	Not available	UAV-aided networks

**Table 3:** Network utilization analysis using boundless area model (kbps).

Metrics	AntHocNet	AOMDV	DSDV	DSR	M-DART	ZRP
Minimum	728.3125	1081.656	797.1563	1608.344	720	720
Maximum	9311.75	4747.359	4019.438	6217.172	4431.688	1320
Average	9311.75	4747.359	4019.438	6217.172	4431.688	1320
Standard deviation	1260.94777	513.0735	405.4626	587.2945	638.467	129.4262

## Data Availability

The data used to support the findings of the study are included within the article.
